The article "Online Algorithm Design of English Translation of Film and Television Works under the Background of Media Cultural Information" was published in 2022. Journal: Comput Intell Neurosci.

# Online Algorithm Design of English Translation of Film and Television Works under the Background of Media Cultural Information

**DOI:** 10.1155/2022/7057322

**Published:** 2022-05-04

**Authors:** JiaXi Sun

**Affiliations:** Chinese Theatre Arts Department, Shandong University of Arts, Shandong, China

## Abstract

As a carrier and medium of culture, film and television have richer cultural connotations and a mission of cross-cultural communication. The translation and dissemination of film and television works not only play an important role in enhancing understanding and communication between different countries, but also contribute to the social life and values of ordinary people. Influence is growing. In order to improve the media communication function of film and television works, this paper attempts to explain and discuss how subtitle translation uses these two translation strategies through the analysis of Chinese and foreign film and television dramas. Through the analysis of the specific translation process of film and television works, the author draws the conclusion that in order to achieve the specific translation purpose, the subtitle translation should be based on the author's intention, translation purpose, text type, and reader factors. This paper adopts a combination of qualitative and quantitative methods and selects suitable examples to explain or illustrate the phenomenon of film and television translation in the description and analysis process. The system designed in the paper is designed with the dissemination and evaluation of film and television works as parameters. The example in this study is that the author himself recorded it according to the Chinese and English subtitles on the screen when watching. Without personal modification, the selected films are officially official institutions, published or broadcast translations. This research focuses on the dialectical analysis and thinking of the collected corpus, so that the conclusions are more convincing than just giving some perceptual examples.

## 1. Introduction

Nowadays, the development of global economy has become the general trend, and the social requirements for the translation industry are also increasing. In addition, English online translation platform (EOTP) and software in the translation field and many unfamiliar with professional features, such as in the field of professional translation for English online translation platform, should be used. In a word, EOTP has good technical support and development prospects, and it will certainly provide more convenient and efficient translation services for various translation needs in the development process.

Today, with the continuous development of the international society, in-depth research on film and television translation can help us understand the real content and deep connotations of films, show the cultural differences between Chinese and English, and further promote cross-cultural communication, understanding, and communication. Today, with the highly developed film and television media, there is not only communication and integration but also fierce competition between film and television cultures in various countries [1]. Therefore, the study of film and television translation increasingly highlights its great significance. The study of film and television translation can greatly promote the communication between Chinese and Western cultures and also conform to the objective requirements of the development of globalization. However, from the perspective of preobjective research, although there are many studies on film and television translation theories in the world, there are few studies on film and television translation from the perspective of norms. From this point of view, this paper will make a more comprehensive and systematic study of film and television translation, so as to better reflect the different characteristics of English and Chinese languages, better convey the real connotation of the film to express, and stimulate people's interest in film and television industry and interest in English and Chinese learning. The study of film and television translation from the perspective of norms can not only narrow the distance between two cultures, but also promote the communication and exchange between different languages and countries [2].

With the rapid development of mobile Internet, as well as the progress of multimedia technology, film and television websites dominated by streaming media service providers emerge and grow. The Internet is becoming the main communication channel of English film and television works in China except cinema and TV [3]. According to statistics from Sohu Video, a domestic streaming media provider, as of November 1, 2014, House of Cards, Season 1, Season 2, Modern Family, Season 1, 234.5 seasons, with English dialogues and bilingual subtitles, have attracted 210 million, 86.98 million, and 304.19 million views, respectively, on Sohu. In September 2014, the author conducted a survey on the movie-watching patterns of 100 college students and 100 IT engineers. IT was found that the frequency of watching English movies through the Internet accounted for 85% and 74% of their total movie-watching in the past three years respectively [4]. IT can be seen that “in terms of workload and job requirements, film and television translation is also one of the most important and fastest growing translations in demand.” English film and television subtitle translation is in full swing, which also promotes the development of domestic subtitle translation research [5]. In contrast, subtitle translation studies in the West “have gradually become part of the central topic” and “have taken a firm foothold in the translation discipline.” “In fact, audio-visual translation research in China is still in its infancy.” For more than a decade, subtitle translation research in China has been mostly confined to the scope of traditional subtitle translation, and insufficient attention has been paid to subtitle translation of English film and television works transmitted on the basis of the Internet, which is inconsistent with the status of the Internet. Therefore, this paper discusses the characteristics and problems of subtitle translation of English film and television works under Internet transmission and puts forward corresponding countermeasures [6].

With the continuous upgrading and development of Internet technology and the continuous advancement of economic globalization, the demand field of translation work is also expanding. English online translation platform is emerging at the historic moment, and it is bound to be in the opportunity period of rapid development in the field of development. However, at present, the major online English translation platforms in the market are all controlled by foreign companies. The scale of Chinese translation platform development companies is small, and the overall industrial concentration is low. The industry as a whole lacks innovation and exploration of technology and model. Currently, English online translation platform development companies generally have two modes of operation: one is the internal production mode combining full-time and part-time translation; the other is the online translation service and business outsourcing model, such as the Domestic Huoyun Translator platform which provides a relatively comprehensive authoritative terminology database to carry out the online translation process between Chinese and English. The user experience of most Online English translation platforms in China is very general, and it is difficult to achieve collaborative management and translation, leading to the progress and efficiency of translation being not up to the best expectation. Meanwhile, most platforms are not compatible with multiple system platforms, which brings a lot of inconvenience to translation work. Except in the field of professional translation, current students to learn English online translation software also has a lot of kinds, such as translation youdao dictionary, Baidu, Google translation, etc., but the development of online translation services function of pure English online translation platform also creates serious development dilemma, especially some free online translation platform. Its rigor, authority, and comprehensiveness need to be improved. Many English online translation platforms cannot provide students with correct translation services, which ultimately affects the quality of learning. At the same time, most online English translation platforms in the market at the present stage lack innovative thinking. The single translation function provided by them will reduce students' ability to explore English learning and make them seriously dependent, which makes it difficult to really improve their English proficiency.

Film and television communication and translation is a large-scale cross-cultural communication activity that follows certain standards and norms. It is a linguistic practice in which content in one language form is reexpressed in another language form. As a modern communication tool, video translation is playing an increasingly important role in today's society, which can be seen from the increasing number of foreign programs introduced and the resulting large number of translation jobs. In Europe, due to the importance attached to film and television translation, many European scholars have written many theoretical works related to subtitle translation, explaining the definition and classification of film and television translation from a theoretical level. For China, the research on film and television translation is still in its infancy, and there is almost no systematic research except for some introductory comments and summaries of practical experience. From a normative point of view, this paper discusses film translation from theory to practice on the basis of some empirical analysis of films, analyzing the problems existing in the field of film translation, the various influencing factors of translation errors by film translators at present, and how to solve the problem of correct translation of film and television works. I hope to bring some highlights and research to film and television translation.

The research contributions of the paper are as follows:

1. This article attempts to explain and discuss how subtitle translation uses these two translation strategies through the analysis of Chinese and foreign film and television dramas.
2. This paper adopts a combination of qualitative and quantitative methods. In the process of description and analysis, appropriate examples are selected to explain or illustrate the phenomenon of film and television translation.
3. The system designed in this paper is designed with the dissemination and evaluation of film and television works as parameters.

## 2. Related Work

At present, film and television translation, as a new field of translation studies, has not attracted enough attention in the field of translation. However, compared with the enormous value and contribution of film and television works to human beings, as well as its impact on human beings, relevant studies on film and television translation are negligible. However, there are also many problems, that is, the lack of a lot of theoretical guidance in film and television translation practice. Western countries, especially Europe, have a relatively early start in the field of film and television translation, with relatively mature theories and relevant systems. In terms of film and television translation, famous scholars at home and abroad have done some relevant studies, which are mainly based on two aspects: foreign and domestic film and television translation studies [7].

At this time, some western scholars began to make some tentative explorations on film and television translation. For example, was published in 1956, and in 1960, by publishing a special edition of Traduction et Cinema, these two articles can master the earliest translation theory studies in the West [8].

Then, in Bable On Subtitles in Television Programmes, Dollerup thought the alphabet study was so important that he undertook a separate alphabet study. In his article, he listed in detail some of the various translation errors commonly seen in TV and movie programs, and the great contribution he made was his research on the teaching significance of alphabet translation. At the same time, he also proposed that subtitle translation of film and television could be used to better promote teaching in English teaching [9, 10].

### 2.1. Design of Network Structure

EOTP can be generally divided into several parts, such as client, server, database, and search engine. It is through these components that the EOTP realizes the connection and exchange of data information, so as to achieve the goal of online translation. The design of network structure is to realize the technology of data exchange, and there are certain differences in different clients.

### 2.2. Design of Hardware and Software System Structure

At the same time, the choice of internal network generally needs to consider many factors, such as platform flow, data throughput, load capacity, operation stability, security, and maintenance cost. Therefore, the hardware architecture of the server should fully consider its load-bearing capacity and operation stability in the process of using. In addition to the consideration of load and security, the development company of English online platform, as a commercial company, has its own commercial purpose, so the design and architecture of hardware mechanism should fully consider the cost performance of server selection and upgrade and maintenance cost. Front-end service software is the realization of information exchange between browser and server. The back-end server is for pretranslation, memory search, term matching and other work, playing the core of the project, processing various business logic [11].

### 2.3. Design of System Functions

After the selection and design of network structure and software and hardware, the EOTP needs to set up functions according to the system requirements. The basic system modules of EOTP based on mobile terminal generally include word query module, single word translation module, new word module, pronunciation module, user management module, and thesaurus management module. Word query translation interface is usually combined by linear and frame methods to realize the multispace attribute of the query interface. There is usually multiple translation result information in the process of query. When the client is connected to the Internet, the word translation module will carry out the process of Chinese-English mutual translation. In the process of word query and translation, if there is no Internet access, the local word database will be searched offline, and then the Chinese-English mutual translation will be carried out. The user management module is an operation module for users to manage software functions [13]. It can delete new words, clear system cache and other functions, and provide software system upgrade and update services. Thesaurus management module provides thesaurus service for users to add words, which is convenient for users to generate exclusive thesaurus according to their own learning conditions, so that they can conveniently use offline query and fast search functions again [12].

## 3. System Design

### 3.1. Hardware Structure Design

The client device is an indispensable hardware device for the online assisted translation system, and it is the main medium for the user to send the HTTP protocol to the server. Without the client, users cannot access the platform, and the translation services provided by different platforms are used.

In general, the following important factors will be fully taken into account in the construction of the internal network of the online assisted translation platform.

1. High load: due to the increasing number of translation company teams and interpreters, the frequency of using online assisted translation platforms will be higher and higher. Therefore, in the server architecture and network design, this will test the load of the server to a great extent.
2. Stability: when the translation company team and translators use the online assisted translation platform, the operation of the system network must be stable enough so that users can enjoy the due convenience.
3. High security: since the online auxiliary translation platform server is built on the public network, anyone anywhere can access the platform as long as they have access to the network. Therefore, the server and firewall of the online translation platform must be able to resist most attacks and viruses on the system from the external network.
4. High cost performance: for server hardware, you can consider renting a server. Use rented servers to deploy our platform applications to achieve a win-win situation.
5. Easy upgrade and maintenance: equipment upgrading and easy maintenance should be taken into account.

If the interpreter wants to export the comparison between the original text and the translation, he/she needs to click the button to download the original text and the translation. The data of the original translation is in the search engine, and the exported text is all Word text. The program flow is shown in Figure 1.

### 3.2. Software Architecture Design

The CSS used on this platform is rendered differently by browser, so it is recommended that you use the Firefox browser to access the platform. Front-end server software: any application that provides HTTP service must have server software. Each server software provides different functional applications, mainly including the network interface module between server and client, Tomcat module, mysql module, and Redis module that provide HTTP request interface. Elasticsearch server module deals with term and memory search, term matching, creation of term database, and memory database. Mysql module handles corpus project domain. This is done for horizontal scaling and security and reliability considerations, preventing the front end from being overstressed.

The leftmost part of the translation interface is the original text area, which contains the translation files uploaded by the interpreter. The translation files are split by the platform into the original text sentence by sentence, which is convenient for the interpreter to translate. The process of splitting sentences and paragraphs of the original text is shown in Figure 2.

### 3.3. Software Functional Module Design

All functional modules of the platform are regarded as a whole, and the modules are first divided into several independent small functional modules according to the hierarchy; then it continues to divide the first layer of submodules by functional modules. Each module should be as independent as possible, and the relationships between modules should be simple and clear, with as few calls and data interactions as possible.

The functional modules of the system are shown in Figure 3.

Each functional module is described as follows.

The basic data maintenance module is used for user authentication, user personal information, and team information identification, which is the main measure to ensure system security and save user data on the platform. Including the realization of the following functional modules.

1. Role management: role management corresponds to the role of interpreters, who are divided into ordinary translators, project managers, and proofreaders. Among them, the project manager can change the basic information of other interpreters, such as the translation language type of the interpreter and the domain type of the interpreter. The interpreter receives the task of translating from the group and adds the glossary. Proofread the documents in real time and inform the relevant translators if there is any problem.
2. Team management: team management includes adding, modifying, and deleting operations. Online auxiliary translation platforms support individual translators while promoting collaborative operations from the team. Translators can only be assigned translation tasks if they join a team. When you sign up for an online assisted translation platform, you have a team, but only you for the time being. Of course you can invite other users to join your team, and you can also join other people's teams.
3. Identity authentication management: when interpreters join a team, they need ID information. Fill in the information necessary to join the team. Through this functional module, the project manager can conveniently manage the team interpreter. When the project manager invites other interpreters to join the team, they do not need to fill in the identification information and can directly join the team invited by the project manager.

The translation module is the working area of the interpreter. It is composed of different areas, and the content presented by the original text area and the translation area is also different. The sentence in the original text area corresponds to a translation in the translation area. In the translation interface, the translator needs to enter the translation into the translation box. If one or some sentences in the memory bank are similar to the current sentence paragraph, they will appear in the translation result area on the right.

1. Source area: after the translation file is uploaded, the system will split the file according to the user-specified format, and the split sentence is the content of the source area. Split format is different, only the number of lines representing the original text area is different, and split format is divided into paragraph, period, character number, and other split methods.
2. Translation area: the translation area is relative to the original area. After translating a sentence, press Enter to save it. The translation area can call the corpus of the search engine for matching.

### 3.4. Translation Design of Film and Television Works

The basic standard can be achieved by limiting the process.

(1) $$\begin{array}{c} \alpha_{i}=\frac{1}{n}\sum_{j=1}^{N_{i}}x_{ij}. \end{array}$$

*x* is the number of words and *N* is the number of nodes, where *α*_*i*_ is the semantic translation context that can be translated, and the selection process of the optimal context *α* is as follows:

(2) $$\begin{array}{c} \alpha_{i}=\frac{1}{K}\sum_{j=1}^{N_{i}}\alpha_{ij}. \end{array}$$

Nonsemantic translation context matrix *S*_*w*_ and suitable semantic translation context matrix *S*_*B*_ are, respectively, calculated as follows:

(3) $$\begin{array}{c} S_{w}=\overset{K}{\underset{i=1}{\sum }}\overset{K_{i}}{\underset{j=1}{\sum }}\left(\alpha_{ij}-\alpha \right){\left(\alpha_{ij}-\alpha \right)}^{K},\\ S_{B}=\overset{K}{\underset{i=1}{\sum }}\left(\alpha_{ij}-\alpha \right){\left(\alpha_{ij}-\alpha \right)}^{k}. \end{array}$$

If *λ* is the optimal context of the semantic context association matrix *S*_*w*_^*T*^*S*_*B*_, and *f* is the criterion to measure the degree of semantic context correlation, the value of *α* can directly reflect the mapping of the correlation process. The semantic context association matrix *S*_*w*_^*T*^*S*_*B*_ has *k* − 1 optimal translation contexts at most, and its optimal contexts are *R*(*R* ≤ *K* − 1):

(4) $$\begin{array}{c} \beta =\left[\alpha_{1},\alpha_{2},\ldots ,\alpha_{R}\right]. \end{array}$$

After the above process, the extraction of the optimal context in the translation process is completed.

Semantically similar words in English-Chinese translation are described as follows:

(5) $$\begin{array}{c} \theta :S⟶S\times \left[-0.5,0.5\right], \end{array}$$

where *θ* refers to the approximate semantics in English-Chinese translation.

(6) $$\begin{array}{c} \Delta :\left[0,T\right]⟶S\times \left[-0.5,0.5\right). \end{array}$$

The interactive English-Chinese translation statements are used for the secondary definition of translation content, which can be expressed as

(7) $$\begin{array}{c} \Delta \left(\beta \right)=\left\{\begin{array}{cc} S_{E}, & K=\text{round}\left(\beta \right),\\ \alpha_{E}=\beta -k, & \alpha_{E}\in \left[-0.5,0.5\right), \end{array}\right) \end{array}$$

where All *F* Match(*M*_*i*_,*M*_*r*_) is the analogical matching function, which can calculate the similarity of structure and components between source language sentence (*M*_*i*_), and pattern library pattern (*M*_*r*_), which is defined as

(8) $$\begin{array}{c} \text{All }F\text{ Match}\left(M_{i},M_{r}\right)=\left\{\begin{array}{cc} 1, & \text{if }M_{i}=M_{r},\\ D\left(M_{i}=M_{r}\right), & \text{if }M_{i}!=M_{r}. \end{array}\right) \end{array}$$

The value range of *D*(*M*_*i*_,*M*_*r*_) is [0,1], indicating the matching difference between *M*_*i*_ and *M*_*r*_. If *M*_*i*_ and *M*_*r*_ are identical, then *D*(*M*_*i*_,*M*_*r*_) has the value 1. If *M*_*i*_ and *M*_*r*_ are completely different, then *D*(*M*_*i*_,*M*_*r*_) has the value 0. When the value of *D*(*M*_*i*_,*M*_*r*_) is between 0 and 1, the closer it is to 1, the greater the matching degree of *M*_*i*_ and *M*_*r*_ is. The closer it is to 0, the smaller the match between *M*_*i*_ and *M*_*r*_ is.

Assuming that CIntra1(*n*) is the association rule set between two nodes in words, phrases or sentences in English literary works, and CInter1(*n*) is the semantic ontology model, then

(9) $$\begin{array}{c} {\text{CIntra}}_{i}\left(n\right)=\frac{{\text{NIntra}}_{i}\left(n\right)}{T},\\ {\text{CInter}}_{i}\left(n\right)=\frac{{\text{NInter}}_{i}\left(n\right)}{T}. \end{array}$$

*T* represents the number of nodes, and *U*_*i*_(*n*) is used to represent the utilization rate of the semantic library, then

(10) $$\begin{array}{c} U_{i}\left(n\right)=\alpha {\text{CIntra}}_{i}\left(n\right)+\left(1-\alpha \right){\text{CInter}}_{i}\left(n\right). \end{array}$$

Let A be the semantic attribute set, B be the semantic category set, and *A* = {*a*_1_, *a*_2_,…, *a*_*n*_}, *B* = {*b*_1_, *b*_2_,…, *b*_*m*_}. The rule set of the relationship between the two is

(11) $$\begin{array}{c} \text{Info}\left(B\right)=-\overset{m}{\underset{i=1}{\sum }}p_{i}\times \;\log_{2}p_{i},\\ {\text{Info}}_{A}\left(B\right)=\overset{v}{\underset{j=1}{\sum }}\frac{\left|B_{j}\right|}{\left|B\right|}\times \text{Info}\left(B_{j}\right),\\ \text{Gain}\left(A\right)=\text{Info}\left(B\right)-{\text{Info}}_{A}\left(B\right). \end{array}$$

Suppose the topological molecular vocabulary of the ontology model is *X* and Y, *C* = {*c*_1_, *c*_2_,…, *c*_*k*_}; then, the association rule vector set of words, phrases, or sentences to be translated is

(12) $$\begin{array}{c} \mathrm{Cos}\left(X,Y\right)=\frac{C\left(X\right)\cdot C\left(Y\right)}{\left|C\left(X\right)\right|\cdot \left|C\left(Y\right)\right|}. \end{array}$$

By analyzing the semantic mapping between *A* and *B*, and then analyzing the eigenvalues of vectors, the complete concept lattice of intelligent translation is constructed.

## 4. Experiment

In this paper, experimental parameters are set, as shown in Table 1.

The experiment designed in this paper requires random selection of experimental objects. In order to ensure the accuracy of the test process, certain conditions are set for the test objects, as shown in Table 2.

Figure 4 is based on feature extraction algorithm designed in this paper, the interactive English Han translation system and the traditional interactive English-Chinese translation system, and section number of control points in the process of translation; on the left side of the translation process of the design of section point distribution diagram, a relatively balanced distribution can be seen from the diagram, the right for the traditional translation of English-Chinese translation system section point distribution; and restrained distribution can reflect the correlation between semantics and context of the translation system. Loose distribution indicates that the translation is correct but lacks contextual coherence. The interactive English-Chinese translation system based on feature extraction algorithm designed in this paper has a compact distribution of translation node control points without loose distribution, indicating that it has a very high translation accuracy.

The comparison of weighted LDA indices is shown in Figure 5.

As can be seen from Figure 5, the weighted LDA indices can be correlated and distributed in an orderly manner, while the translation results of traditional English-Chinese translation systems are obviously lacking of the relationship between the weighted LDA indices and the weighted LDA indices. Unweighted LDA index is a measure of semantic depth connection in the process of translation. When weighted LDA indexes are connected together in order, it indicates that the translation process is vivid and deep; when weighted LDA indexes are scattered, it indicates that the focus of translation semantics is not grasped.

## 5. Conclusion

In order to study the dissemination of film and television works, this paper analyzes the translation of film and television works from multiple perspectives based on normative principles. Through the analysis of some film and television works, this paper discusses film translation from theory to practice and analyzes the problems existing in the field of film translation. Now, the various influencing factors of translation errors by film translators and how to correctly translate film and TV works are hoped to give the study of film translation some enlightenment, which provides a good reference for future film translation. Due to the author's computer software technology and limited time, the platform also has some defects, and users cannot upload project files in DWG or DXF format. At the same time, translation is a big topic, and online assisted translation platforms only solve a small part of the translation industry. With the emergence of new computer technologies and improvements in computer hardware, the author will continue to improve translation platforms. In the future research process, how to conduct regular research on different film and television works will be a research focus.

## Figures and Tables

**Figure 1:** Export the original text and the translation comparison.

**Figure 2:** Separation flow chart of the original text.

**Figure 3:** System function module diagram.

**Figure 4:** Results of comparison test.

**Figure 5:** Results comparison of different English-Chinese translation systems. (a) Traditional systems. (b) Improved system.

**Table 1:** Test parameters.

The basic parameters	Value
Phrase translation quantity/character	300
Short passage translation per word	450
Translation rate/(kbit/s)	12
Semantic recognition rate/(kbit/s)	20

**Table 2:** Setting of test data.

Number of test	Type of contextual translation	Comprehensive revision parameter
1	2	0.1 × 10^−3^
2	3	0.2 × 10^−3^
3	2	0.1 × 10^−3^
4	3	0.2 × 10^−3^
5	2	0.1 × 10^−3^
6	3	0.2 × 10^−3^

## Data Availability

The data used to support the findings of this study are available from the corresponding author upon request.
